The article "Successful treatment of idiopathic mast cell activation syndrome with low‐dose Omalizumab" was published in 2019. Journal: Clin Transl Immunology.

# Successful treatment of idiopathic mast cell activation syndrome with low‐dose Omalizumab

**DOI:** 10.1002/cti2.1075

**Published:** 2019-09-30

**Authors:** Renee Berry, Peter Hollingsworth, Michaela Lucas

**Affiliations:** ^1^ Department of Clinical Immunology Sir Charles Gairdner Hospital Nedlands WA Australia; ^2^ Path West Queen Elizabeth II Medical Centre Nedlands WA Australia; ^3^ Medical School University of Western Australia Nedlands WA Australia

**Keywords:** bee venom immunotherapy, idiopathic non‐clonal mast cell disorder, mast cell activation syndrome, omalizumab

## Abstract

**Objectives:**

Idiopathic mast cell disorders, a recently defined and recognised syndrome in clinical practice, are similar to the previously termed non‐clonal mast cell disorder. Patients with idiopathic mast cell activation syndrome (MCAS) suffer all the classical signs of mast cell activation but do not have evidence of mast cell clonality. Furthermore, treatment of these patients can be limited and burdensome in those with refractory symptoms.

**Methods:**

Here, we describe treatment of a patient with idiopathic MCAS utilising a single monthly subcutaneous injection of omalizumab and review the current classification and therapeutic options for clonal and non‐clonal MCAS.

**Results:**

Low‐dose omalizumab treatment has successfully led to a 5‐year, sustained clinical response, controlled debilitating symptoms of mast cell activation and allowed for reintroduction and long‐term maintenance of bee venom subcutaneous immunotherapy.

**Conclusion:**

Low‐dose omalizumab of 150 mg monthly should be considered for maintenance management of patients with idiopathic MCAS for its cost and quality‐of‐life benefits.

## Case report

Our case, a 48‐year‐old man, presented in January 2011 after suffering a road traffic accident. This occurred following anaphylaxis with complete loss of consciousness while driving, 15 min after being stung by a bee. He had previously experienced large local reactions to bee stings but no anaphylaxis. Past medical history was of avocado oral food allergy, with no other significant history of allergies, and TIA secondary to the presence of a patent foramen ovale for which he was on aspirin. This episode was not associated with any focal neurology, rash or respiratory symptoms and responded rapidly to 500 μg of intramuscular adrenaline. Baseline serum mast cell tryptase (MCT) was 19.2 μg L^−1^ (Figure 1; normal< 14.0 μg L^−1^) and serum immunoglobulin E 344 kU L^−1^ (normal < 111 kU L^−1^). Bee venom‐specific IgE was 60.5 kU L^−1^ (very high > 17.5 kU L^−1^) and avocado 6.84 kU L^−1^ (high > 3.5–17.5 kU L^−1^). He commenced bee venom subcutaneous allergen immunotherapy (BV‐SCIT) in February. Six months into BV‐SCIT on a maintenance dose of 100 μg bee venom extract, he suffered an allergic reaction. Symptoms appeared within minutes of receiving the injection, including alteration in vision, generalised malaise, light‐headedness and the fear of impending collapse. The symptoms resolved with administration of 500 μg of adrenaline intramuscularly. In September 2011, BV‐SCIT was recommenced and continued at 100 μg per month until the beginning of August 2013 when he suffered another reaction. He was pale and unwell with a sensation of light‐headedness and impending loss of consciousness. He was treated for anaphylaxis and improved after 500 μg adrenaline injection; however, the reaction continued for 30 min despite a second adrenaline injection 20 min later. He was observed in the emergency department and further treated with 100 mg IV hydrocortisone and intravenous fluids and discharged after a five‐hour period of observation. One week later, he was admitted to hospital for persistent symptoms of light‐headedness and impeding collapse. He was commenced on regular Prednisolone 25 mg daily and cetirizine 10 mg twice daily. During his admission, he was noted to have a significant postural blood pressure drop of 40 mmHg, which was followed by a 20‐min episode of severe lower abdominal pain. MCT level was 18.0 μg/L. Hypoglycaemia, myocardial infarction, pulmonary embolism and infection were excluded with normal serum blood glucose, troponin, CK, d‐dimer and CRP on laboratory tests. Serum fractionated catecholamines and metanephrines testing for pheochromocytoma and urinary 5‐HIAA testing for carcinoid were negative. Dermatological examination excluded cutaneous mastocytoma. Bone marrow aspirate revealed normal trilineage haematopoiesis with no increase in mast cell numbers. Molecular testing for c‐KIT D816V in marrow and serum was negative. The bone marrow trephine staining for CD2 and CD117 did not demonstrate a significant mast cell population. Despite a persistently elevated kappa/lambda ratio of 2.44, serum protein electrophoresis was negative for monoclonal immunoglobulins and full‐body PET scan revealed no area of abnormal scintigraphic uptake. Notably, bone mineral density completed before the commencement of Prednisolone determined a T score of −1.5 at the spine which was low normal in comparison with the young adult reference population. Treatment montelukast 10 mg in combination with thrice‐daily cetirizine 10 mg or fexofenadine 180 mg was commenced after discharge in addition to the Prednisolone. Prednisolone was then weaned over 6 months and ceased in April 2014. Despite treatment, his symptoms progressed. He further described mental clouding, poor concentration and early morning wakening. By July 2014, he reported daily symptoms of impending collapse especially with exercise and a reduced tolerance to red wine and caffeine. Consequently, he decided to resign from his employment as a Chief Executive Officer and seek management from a clinical psychiatrist to manage anxiety and depressive symptoms. The combination of symptoms, persistently elevated MCT and negative bone marrow testing led to the diagnosis of non‐clonal MCAS and advised to avoid food rich in tyramine and histamine and to limit any strenuous exercise. There was minimal symptomatic improvement. Omalizumab, rather than an alternate mast cell stabiliser, was commenced in October 2014 because of persistent and severe symptoms at 150 mg, two doses 1 week apart, to allow for the recommencement of BV‐SCIT. Using a rapid up‐dosing protocol, BV‐SCIT was re‐initiated 2 weeks later (Table 1). Since that time, he reports improved mental clarity, reduction in anxiety symptoms and overall general improvement in health, allowing him to return to his work. By choice, he continues a histamine‐free diet but can freely complete any cardiovascular exercise. Omalizumab has been well tolerated, the only reaction occurring following the initial 150 mg injection where he reported pre‐syncopal symptoms and a recorded bradycardia of 40 bpm. He has been able to reduce his daily use of antihistamines to one tablet of fexofenadine (180 mg) in addition to 10 mg montelukast (Figure 1). He no longer requires Prednisolone. Triggers such as exercise, emotional stress and spicy foods which were initially major contributors to symptoms now do not cause exacerbations. He receives monthly doses of subcutaneous 150 mg omalizumab along with maintenance BV‐SCIT at 100 μg. Mast cell tryptase levels remain stable, albeit elevated (Figure 1).

The article "Successful treatment of idiopathic mast cell activation syndrome with low‐dose Omalizumab" was published in 2019. Journal: Clin Transl Immunology.

**Figure 1:** Mast cell tryptase (MCT) level with the progression of symptoms and events over a 5‐year period. Despite current elevations of MCT >19.5 μg L^−1^ in June 2016, the patient remains symptom‐free with maintenance 150 mg omalizumab monthly and ongoing maintenance BV‐SCIT. ^Omalizumab induction regime 150 mg, two doses, 2 weeks apart. *Reduced doses of antihistamines required with the introduction of omalizumab. Cetirizine 30 mg daily reduced to 10 mg daily and fexofenadine 720 mg daily to 180 mg daily. Prednisolone 50 mg weaned to 5 mg and then ceased.

**Table 1:** Bee venom subcutaneous immunotherapy protocol utilised in this patient

Day	Concentration (μg mL^−1^)	Volume (mL)	Dose (μg)
1	0.1	0.1	0.01
1	1	0.1	0.1
1	1	0.5	0.5
1	10	0.1	1
1	10	0.2	2
8	1	0.1	0.1
8	10	0.1	1
8	10	0.5	5
8	100	0.1	10
8	100	0.2	20
15	100	0.3	30
15	100	0.3	30
15	100	0.3	30
22	100	1.0	100
36	100	1.0	100
57	100	1.0	100
Four weekly	100	1.0	100

Following each injection, wheal and flare is documented, as well as the presence of any systemic reactions prior to proceeding to the next step. The final four‐weekly dosing of BV‐SCIT is 100 μg given as split dosing 30 min apart. 150 mg omalizumab subcutaneous injection is given 30 min prior to the bee venom administration, at the four‐weekly interval.

## Differential diagnosis

As reviewed by Akin^1^, ^2^ subsequently Hamilton^3^ and most recently Valent *et al*.,^4^ mast cell activation syndromes have been divided into primary, secondary, idiopathic and non‐clonal. Based on our patient's symptoms and the current classification system, a diagnosis of idiopathic non‐clonal mast cell activation syndrome has been made (Table 2). Suggestion of the familial nature of mast cell disorders is evidenced by his son being found to also have an elevated serum MCT of 16.5 μg L^−1^ without clinical symptoms. Our patient does not meet the current diagnostic guidelines for monoclonal mast cell activation disorder due to the lack of cKIT mutation in serum and bone marrow and lack of clonal CD2 mast cell staining. The mast cell tryptase level has been elevated for 5 years without emergence of a definite primary mast cell disorder (systemic or monoclonal). This patient also does not align the diagnosis of a secondary mast cell activation disorder as we have excluded lymphoproliferative disease, infection and significant atopic disease and mast cell morphology is immature. Finally, the diagnoses of idiopathic anaphylaxis are less likely, as the patient does not show signs of clear and intermittent mast cell degranulation, and without return of his mast cell tryptase level to normal baseline. In this context, he also lacks clinical cutaneous and respiratory symptoms, commonly seen in anaphylaxis.

**Table 2:** Common features of mast cell activation syndromes and comparative phenotypic features of our patient (+ present in our patient and − absent in our patient) with idiopathic non‐clonal mast cell activation syndrome. Refer to references for complete definitions [1–4]

MCAS	Typical features	Our patient
Primary		
Mastocytosis	Kit D816V mutation	−
Monoclonal mast cell activation disorders	Aberrant CD25+/−CD2 staining	−
	Urticaria	−
	Anaphylaxis/syncope	+
	Bee venom allergy	+
Secondary		
Allergic disorders	Elevated serum‐specific IgE	+
Physical urticaria	IgE‐mediated allergy	+Bee venom
Mast cell activation with chronic inflammation	Non‐IgE‐mediated allergy	+Exercise and psychological
	Infection	−
	Lymphoproliferative disease	−
	Autoimmunity	−
	Mature mast cell histology	−
Idiopathic		
Anaphylaxis	Female sex^a^	−
Urticaria	Cutaneous symptoms	−
Histaminergic angioedema	Respiratory symptoms	−
Mast cell activation syndrome	Good response to mast cell stabilising medications	−
	Return to baseline MCT	−

IgE: immunoglobulin E; MCAS: mast cell activation syndrome; MCT mast cell tryptase.

a Commonly idiopathic urticaria now known as chronic spontaneous urticaria.

The article "Successful treatment of idiopathic mast cell activation syndrome with low‐dose Omalizumab" was published in 2019. Journal: Clin Transl Immunology.

## Comments

This patient presents with a MCAS, best defined as an idiopathic non‐clonal MCAS.^5^ Recurrent mast cell activation was evidenced by his clinical symptoms, notable reduction in bone mineral density on radiological investigations and ameliorated by low‐dose omalizumab therapy. Omalizumab works to block the binding of free IgE to its corresponding FcεRI receptor on basophils and mast cells consequently inhibiting their activation by allergens; thus, omalizumab can act as a basophil and mast cell stabiliser. The improvement in our patient's symptoms on low‐dose omalizumab therapy points towards possible aberrant mast cell FcεRI activation in the underlying pathogenesis of this patient's symptoms. The likely mechanism involves downregulation of mast cell FcεRI receptors and the reduction in release of pro‐inflammatory cytokines preventing downstream allergic inflammation and hypersensitivity reactions.^6^ Omalizumab is generally well tolerated with infrequently reported adverse reactions including local injection site reactions and headache. Less commonly reported reactions include musculoskeletal (arthralgias, myalgias), skin (pruritus, urticaria) and respiratory (nasopharyngitis, sinusitis), with few case reports of anaphylaxis occurring up to 1 year postcommencement of treatment. A recent prospective study of 56 patients with a range of mast cell diseases, including 11 patients with idiopathic mast cell disorder (confirmed KIT mutation‐negative), has further described the benefit of omalizumab therapy, notably for the relief of vasomotor symptoms and recurrent anaphylaxis as well as moderate improvements in neuropsychiatric symptoms with an associated favorable safety profile.^7^ In this study, the dosing schedule was at least double the dose with a minimum of 300 mg per month up to 1200 mg per month. Further cases of omalizumab treatment in primary/monoclonal MCAS have also been summarised recently by Jagdis and Vadas^8^ and Bell and Jackson.^9^ To our knowledge, this is the first case where very low‐dose (150 mg) monthly omalizumab injections have successfully led to a 5‐year, sustained clinical response and controlled debilitating symptoms allowing for maintenance BV‐SCIT in an adult with idiopathic MCAS. Thus, low‐dose omalizumab can have a sufficient mast cell stabilising effect. It, therefore, should be considered for the long‐term management of patients with MCAS for its cost–benefit as well as reduction of frequency of injections and medical visits for the patient.

The article "Successful treatment of idiopathic mast cell activation syndrome with low‐dose Omalizumab" was published in 2019. Journal: Clin Transl Immunology.

## Conflict of Interest

There are no conflicts of interest.
